RETRACTED

# Isolation of a Reassortant H1N2 Swine Flu Strain of Type “Swine-Human-Avian” and Its Genetic Variability Analysis

**DOI:** 10.1155/2018/1096079

**Published:** 2018-05-29

**Authors:** Long-Bai Wang, Qiu-Yong Chen, Xue-Min Wu, Yong-Liang Che, Cheng-Yan Wang, Ru-Jing Chen, Lun-Jiang Zhou

**Affiliations:** Institute of Animal Husbandry and Veterinary Medicine, Fujian Academy of Agriculture Sciences, Fujian Animal Disease Control Technology Development Center, Fuzhou, Fujian 350013, China

## Abstract

We isolated an influenza strain named A/Swine/Fujian/F1/2010 (H1N2) from a pig suspected to be infected with swine flu. The results of electron microscopy, hemagglutination (HA) assay, hemagglutination inhibition (HI) assay, and whole genome sequencing analysis suggest that it was a reassortant virus of swine (H1N1 subtype), human (H3N2 subtype), and avian influenza viruses. To further study the genetic evolution of A/Swine/Fujian/F1/2010 (H1N2), we cloned its whole genome fragments using RT-PCR and performed phylogenetic analysis on the eight genes. As a result, the nucleotide sequences of HA, NA, PB1, PA, PB2, NP, M, and NS gene are similar to those of A/Swine/Shanghai/1/2007(H1N2) with identity of 98.9%, 98.9%, 99.0%, 98.6%, 99.0%, 98.9%, 99.3%, and 99.3%, respectively. Similar to A/Swine/Shanghai/1/2007(H1N2), we inferred that the HA, NP, M, and NS gene fragments of A/Swine/Fujian/F1/2010 (H1N2) strain were derived from classical swine influenza H3N2 subtype, NA and PB1 were derived from human swine influenza H3N2 subtype, and PB2 and PA genes were derived from avian influenza virus. This further validates the role of swine as a “mixer” for influenza viruses.

## 1. Introduction

Swine influenza is an acute and highly contagious flu caused by swine influenza virus (SIV), which infects human and pigs. Its clinical symptoms in swine include high fever, decreased appetite, lethargy, sneezing, coughing, and difficulty in breath [1]. In virus classification, swine influenza viruses are single-stranded negative-sense RNA viruses belonging to the family Orthomyxoviridae. The genome of swine influenza virus is composed of 8 gene fragments with different sizes, namely, PB2, PB1, PA, HA, NP, NA, M, and NS, respectively [2]. The 8 genomic segments of different influenza viruses can be randomly shuffled to generate new reassortant viruses [3]. As pigs possess both NeuAc-2,3Gal and NeuAc-2,6Gal receptors, they can infect both human and avian influenza viruses [3]. As a result, pigs become a “mixer” for reassortment of influenza viruses and an “incubator” for emergence of new influenza strains [4, 5]. Pigs also play an important role in the ecological distribution and genetic evolution of influenza viruses. For example, the Sydney-like H3N2 mutant isolated in the United States in 1998 is an “avian-swine-human” reassortant strain [6]. In addition, the pandemic H1N1 influenza virus originated in April 2009 is a “swine-human-avian” reassortant virus [7]. In fact, two out of the four most serious influenza pandemics in the history are caused by reassortment of gene segments from avian influenza viruses [8, 9].

RETRACTED

At present, there are three subtypes of swine influenza in the world, namely, H1N1, H3N2, and H1N2, which can be further divided into classic swine H1N1, avian H1N1, human-like H3N2, reassortant H3N2, and reassortant H1N2 [10, 11]. In addition to these three subtypes, strains of subtypes H5N1, H9N2, and H3N1 have also been isolated in swine populations; however they are not prevalent enough in swine populations to establish stable lineages [12–14]. The H3N2 swine influenza subtype was first reported in Taiwan in 1969, and the H3N2 swine influenza viruses were isolated from pigs in Hong Kong in 1970 [15]. After that, they have become widespread in swine worldwide. H1N2 influenza subtype was first isolated from Japanese swine herds in 1978 and subsequently widespread in other countries such as France, UK, and USA. The H1N2 swine influenza viruses are diverse in gene origin, which results in their different levels of prevalence and danger. In China, H1N2 swine influenza virus was first isolated in Zhejiang in 2004 and then isolated in Guangxi, Shanghai, Guangdong, and other places from 2005 to 2010.

From 2009 to 2013, our laboratory carried out epidemiological study of swine flu in Fujian Province. An influenza strain was isolated from 13 pigs suspected to be infected. We then performed electron microscopy, hemagglutination (HA) assay, hemagglutination inhibition (HI) assay, and whole genome sequencing analysis to infer its biological characteristics and evolutionary history. As a result, we confirmed that the virus was a “swine-human-avian” reassortant virus.

## 2. Materials and Methods

### 2.1. Materials

*Materials and Reagents. *The lungs and lymph nodes used in the experiment were collected from a large-scale swine farm suspected to be infected with swine influenza in Fujian Province, China. EDS-76 and ND were positive sera provided by Fujian Institute of Animal Husbandry and Veterinary Medicine; the standard antigens and its antisera of H1, H3, H5, H7, and H9 subtypes and antisera of N1, N2, and N9 subtypes were purchased from Harbin Veterinary Research Institute; RNA extraction kit Trizol, plasmid extraction kit, LATaq DNA polymerase, RNasin Inhibition, M-MLV, dNTP, BamHI, HindIII, and PMD18-T vector were purchased from Dalian Bao Biological Company;* Escherichia coli* engineering strain DH5a was preserved by our laboratory.

RETRACTED

*Test Animals*. BALB/c mice were collected from Fujian Medical Laboratory Animal Center; 5-week-old piglets were purchased from a large-scale pig farm in Fuzhou, which were confirmed to be negative in serological antibody examination; SPF eggs were purchased from Fuzhou Dabei Agricultural Biotechnology Co. and incubated to 9 to 11 days of age.

### 2.2. Virus Isolation

*Acquisition and Processing of Disease Materials*. The lung and lymph node tissues of pigs suspected to be infected with swine influenza were cut into pieces and ground into homogenate under sterile conditions. Hank's solution was added to it to make 10% suspension solution, which was then undergone frozen and thawed for three times, centrifuged at 12000 rpm for 10 min. The supernatant was filtered and sterilized, and placed at −70°C freezer for further use.

*Virus Isolation and Culture*. The supernatant was inoculated into allantoic cavity of 9 to 11-day-old SPF chicken embryos with 0.1 mL/embryo, and each sample was inoculated into 4 embryos. The inoculated embryos were incubated in an incubator at 37°C and a relative humidity of 55%. The eggs were candled twice a day to inspect the vitality of chicken embryos for 6 days. The embryos died within 24 hours were abandoned, whereas those died between 24 and 96 hours were stored overnight at 4°C. Allantoic fluid was collected and the hemagglutination activity was detected. If the hemagglutination result is positive, we preserved chicken embryo allantoic fluid; otherwise the allantoic fluid were blindly passed for three generations and discarded if the result was still negative.

### 2.3. Virus Identification

*Swine Influenza RT-PCR*. A pair of primers was designed according to the M gene conserved region of swine flu registered in GenBank, i.e., SIV-F: 5′-CAAGACCAATCCTGTCACCTC-3′, and SIV-R: 5′-AAGACGATCAAGAATCCAC AA-3′. It was then amplified into a fragment of 684 bp by synthetic company Dalian Biological Engineering Technology. The viral RNA was extracted by conventional methods. The 10.0 *μ*L RT reaction system consists of DEPC water (1.25 *μ*L), 5 × AMV Buffer (2.0 *μ*L), 25 mg MgCl_2_ (1.0 *μ*L), dNTP mixture (1.0 *μ*L), RNase inhibitor (0.25 *μ*L) of AMV (0.5 *μ*L), random primer (1.0 *μ*L), and RNA sample template (3.0 *μ*l). The RT reaction conditions were 30°C for 10 min, 42°C for 1 h, and 99°C for 5 min. The 25.0 *μ*L PCR reaction system consists of Nuclease-Free Water (10.0 *μ*L), GoTaq Green Master Mix (10.0 *μ*L), upstream primer (0.5 *μ*L), downstream primer (0.5 *μ*L), and RT reaction product (4.0 *μ*L). The PCR reaction conditions were 95°C for 5 min, 94°C for 1 min, 54°C for 1 min, 72°C for 1 min with 35 cycles, and then 72°C for 10 min and 4°C for preservation. After the reaction, the PCR products were electrophoresed on 1% agarose gel, and the positive product was sequenced by Bioengineering (Shanghai) Co., Ltd.

RETRACTED

*Electron Microscopy*. After allantoic fluid was centrifuged by differential and density gradient method, the morphology and size of the virus were observed by transmission electron microscopy.

*Agar Diffusion Test*. The isolated chicken embryo allantoic fluid was purified, which can be used as antigen after adding SDS. After that, it was under agar diffusion test with standard serum. The results were collected at 24 h, 48 h, and 72 h, respectively.

### 2.4. Identification of Serum Subtypes

The HA subtype of swine influenza virus was identified by comparing the isolated virus with the standard positive sera of swine influenza by hemagglutination assay (HA) and hemagglutination inhibition assay (HI). Neuraminidase inhibition assay (NI) was used to identify NA subtypes.

*Hemagglutination Assay (HA)*. We added 50 *μ*l of virus antigen in the first well of each row and used a pipette to mix well; we then added 50 *μ*l of the mixed solution to the second well, diluted consecutively until the 11th well. The 12th hole without antigen was taken as a control. After that, we added 50 *μ*l 1% pigeon erythrocyte suspension to each well, oscillated using microoscillator for 1 min and recorded the results after 20 ~ 30 min quiescence in room temperature.

*Hemagglutination Inhibition Assay (HI)*. According to the hemagglutination test, we made 8-unit and 4-unit antigen by adding physiological saline. We then added 50 *μ*l 8-unit antigen into the first well and 50 *μ*l 4-unit antigen into the 2nd, 3rd,…, and 11th well and 50 *μ*l normal saline to the 12th well as negative control. After that, we took 50 *μ*l standard positive serum to the first well, mixed them even, and took 50 *μ*l to the second well. The process was repeated until the 11th well. After 15 min at room temperature, we added 50 *μ*l 1% pigeon erythrocyte suspension, oscillated using microoscillator for 1 min and recorded the results after 20 min quiescence in room temperature. The hemagglutination inhibition titer of the serum was the maximum dilution of sera with 50% inhibition of erythrocyte agglutination. Hemagglutination inhibition titer ≥ 4log3 serum was determined as positive.

*Neuraminidase Inhibition Assay (NI)*. The allantoic fluid of the virus was tested against the standard antiserum of three NA subtypes.

### 2.5. Half of the Chicken Embryo Infection Determination

The virus liquid of each dilution was inoculated into 9-day-old SPF chicken embryos with 4 pieces/group and 0.1 mL/piece. The embryos were then sealed with wax and cultured at 37°C for 7 days. The embryos which died within 24 hours were abandoned and allantoic fluid from embryos which died after 24 hours were collected for hemagglutination assay and the EID_50_ was calculated by Karber's method.

RETRACTED

### 2.6. Identification of Viral Physical and Chemical Characteristics

Virus allantoic fluid was centrifuged at 3000 rpm for 15 min, and the supernatant was distributed into several tubes for further use. We then added SDS (1 mg/mL, pH 8.2 for 1 h), chloroform (final concentration 48 mL/L at 4°C for 10 min), ether (final concentration 200 mL/L at 4°C for 24 h), hydrochloric acid (final concentration 1 mL/L for 3 min), 1% potassium permanganate (for 5 min), formaldehyde (final concentration 0.2%), and 75% ethanol (for 5 min) and treated them with water at 56°C for 0,5, 10,15, 20, 30, 60, 90, 120, and 180 mins overnight. The treated virus was inoculated into 9-day-old SPF chicken embryo with 0.1 mL/embryo. Allantoic fluid or the embryo died in 24 ~ 96 h were collected for HA assay.

### 2.7. Animal Vaccination Test

*BALB/c Mice Infection Assay*. The virus with the dose 2 × 10^5^EID_50_ was inoculated intranasally into ten 6-week-old BALB/c mice and physiological saline was inoculated into 10 mice as controls. One BALB/c mouse was dissected on the 1st, 3rd, 5th, 7th, 9th, 11th, and 13th days after inoculation. The lungs were harvested for virus isolation. The mental and diet status of the mice were also observed for 2 weeks.

*Infection Assay on Piglets*. Twelve 5-week-old piglets, which were tested negative for swine influenza virus, were divided into experiment and control group evenly. Piglets in experiment were inoculated intranasally with 2 × 10^6^EID_50_ dose viruses and those in control group were inoculated with normal saline. The body temperature of all piglets was measured every day after inoculation, and the diet and mental status of piglets were observed continuously for 28 days.

### 2.8. Whole Gene Sequencing

*Primer Synthesis*. According to the H1N2 subtype of swine influenza virus in GenBank, 12 pairs of primers containing 8 gene fragments were designed by oligo 6.0 software. The primers were available upon request.

*Virus RNA Extraction and RT-PCR Reaction*. Total RNA was extracted from the viral RNA extraction kit Trizol. The RT reaction conditions were DEPC water (1.25 *μ*L), MgCl2 (1.0 *μ*L), 5 × MMLV Buffer (2.0 *μ*L), dNTP Mixture (1.2 *μ*L), MMLV (0.5 *μ*L), RNase Inhibition (0.25 *μ*L), Uni-12 primer (1.0 *μ*L), RNA (3.0 *μ*L); the reaction conditions were 30°C for 10 min, 42°C for 60 min, and 99°C for 5 min and preserved at 4°C. The PCR reaction conditions were 10× PCR Buffer (2.0 *μ*L), dNTP Mixture (1.2 *μ*L), DNA polymerase (0.2 *μ*L), Up Primer (0.4 *μ*L), Down Primer (0.4 *μ*L), and template (2.0 *μ*L) and filled to 20 *μ*L by adding H_2_O. The reaction conditions were as follows: predenaturation at 95°C for 5 min, denaturation at 94°C for 1 min, annealing at 53.5-61.0°C for 1 min, extension at 72°C for 1 min, and extension at 72°C for 10 min. The PCR products were identified by 1.0% agarose gel electrophoresis

*Gene Cloning and PCR Identification*. The PCR product was ligated into PMD18-T vector and transferred into DH5*α* strain. The recombinant plasmid was identified by 1.0% agarose gel electrophoresis, and the positive plasmid was sent to Bioengineering (Shanghai) Co., Ltd., for sequencing.

RETRACTED

### 2.9. Comparison of Gene Sequence Analysis

The sequences were put into GenBank for homology search using BLAST, and the sequences of subtypes human influenza H3N2, swine flu H3N2, classical swine flu H1N1, and representative swine flu H1N2 were downloaded and analyzed by DNAStar software. The sequence alignments were done by MUSCLE software in MEGA6 (http://www.megasoftware.net/). The phylogenetic trees were generated using the Neighbor-Joining method with 1000 bootstrap replicates.

## 3. Results

### 3.1. Virus Isolation

We collected allantoic fluid from inoculated SPF chick embryos died between 24 to 72 hours, whose hemagglutination titer was determined to be 2^5^. By autopsy, we found that there are serious embryo hemorrhage lesions.

### 3.2. Virus Identification

RT-PCR amplification products were detected by agarose gel electrophoresis (Figure 1). As can be seen, the amplified fragments are of sizes about 684 bp as expected. Sequence analysis showed that the gene fragment was derived from swine flu. By visualizing allantoic fluid after centrifugation using electron microscope, one can find influenza virus particles of diameter 80 ~ 120 nm. They are in spherical, horseshoe-shaped, and filamentous enveloped shapes (see Figure 2).

There are white precipitate line identified in the agar diffusion assay between tested antigen and standard influenza A serum, indicating that the isolated virus was an influenza A virus. We then performed HI assay between allantoic fluid and standard positive sera of EDS-76 and ND. The results showed that the isolated strain cannot be inhibited by both EDS-76 and ND, indicating that it is not an EDS or NDV virus. We also performed HA and HI assay against the standard serum of H1 subtype and showed that it can be inhibited by H1 serum with HI value 8 log2, suggesting that the hemagglutinin of the virus is of H1 subtype. In addition, the NI assay suggested that the neuraminidase of the virus is of subtype N2. As a result, we named the virus A/Swine/Fujian/F1/2010 (H1N2). Finally, the EID_50_ value of the fourth-generation allantoic fluid isolated from culture was 10^−4.6^/0.1 mL. The virus lacks resistance to SDS, chloroform, ether, hydrochloric acid, 1% potassium permanganate, formaldehyde, and 75% ethanol and can easily be inactivated. The titer of hemagglutination decreased by 2 titers at 56°C for 5 min. According to the method of determining the thermal stability, it can be determined that the virus strain is heat-labile.

RETRACTED

### 3.3. Animal Vaccination

We first performed BALB/c mouse infection assay. The mice in the experiment group showed symptoms of mental exhaustion, coarse coat, and dyspnea symptoms 3 days after inoculation, but no mice died. The control group was normal. Influenza virus was isolated from the lungs of mice from 1 to 5 days after inoculation, and no virus could be isolated after 7 days after inoculation.

We then infected virus with 6-weed-old piglets. Similar to mice, piglets in experiment group developed symptoms of high body temperature, loss of appetite, cough, and runny nose after 4 days of inoculation, and the symptoms were relieved after 7 days until all the piglets were recovery. No piglets died in the process. In contrast, piglets in control group were normal.

### 3.4. Whole Genome Sequencing and Genetic Variation Analysis

The PB2, PB1, PA, HA, NP, NA, M, and NS genes of A/Swine/Fujian/F1/2010 (H1N2) strain were amplified by RT-PCR, respectively. After sequencing, we obtained 2341 bp, 2302 bp, 2190 bp, 1709 bp, 1543 bp, 1443 bp, 991 bp, and 882 bp gene fragments (Figure 3), which were uploaded to NCBI with accession numbers KM186312, KM186311, KM186310, KM186305, KM186308, KM186307, KM186306, and KM186309, respectively.

We then performed nucleotide homology and genetic phylogenetic analysis using BLAST (https://blast.ncbi.nlm.nih.gov/Blast.cgi), DNAStar (https://www.dnastar.com/), and MEGA6 using Neighbor-Joining method with 1000 bootstrap replicates. We used K80 model to estimate the distances between nucleotides. Specifically, the eight gene fragments of A/Swine/Fujian/F1/2010 (H1N2) strain were compared with human influenza, avian influenza, and swine influenza virus deposited in NCBI flu database.

The nucleotide sequences of HA, NA, PB1, PA, PB2, NP, M, and NS genes all had the highest homology with A/Swine/Shanghai/1/2007 (H1N2) with identity 98.9%, 98.9%,99.0%, 98.6%, 99.0%, 98.9%, 99.3%, and 99.3%, respectively. According to the phylogenetic tree, the HA, NA, PB1, PA, PB2, NP, and M gene fragments of A/Swine/Fujian/F1/2010 (H1N2) is genetically close to those of A/Swine/Shanghai/1/2007(H1N2), while its NS fragment is close to A/Swine/Guangxi/13/2006 (H1N2). We illustrated the phylogenetic trees of HA, NA, PB1, PA, and PB2 in Figures 4–8, respectively.

RETRACTED

### 3.5. Analysis on the Sources of Gene Fragments

The analysis of 8 gene fragments of A/Swine/Fujian/F1/2010 (H1N2) strain showed that the HA, NP, M, and NS gene fragments were originated from classical pig influenza H3N2 subtype, NA and PB1 were derived from human swine influenza H3N2 subtype, and PB2 and PA gene were from avian influenza virus, as shown in Figure 9. The results indicated that the strain was a “swine-human-avian” reassortant virus.

## 4. Discussion

Swine as a host of influenza virus can simultaneously infect different types and subtypes of influenza viruses. Therefore, most scholars believe that swine plays an important role in influenza pandemic as a “mixer” of virus reassortment [2]. When pigs infect both human and avian influenza viruses at the same time, new strains may be produced due to gene reassortment, causing epidemics. The southern part of China is considered to be the source of the world's flu outbreak due to its unique ecological, geographical, and climatic conditions. Fujian locates in southern China, next to Guangdong, one of the most frequent influenza out-breaking places in the world. There are a lot of pig farms and waterfowl habitats in Fujian, greatly increasing the chance of influenza virus reassortment.

Currently, there are a lot of reports about swine influenza virus reassortment all over the world. For example, the H3N2 reassortant virus is isolated from North Carolina in 1998, whose HA, NA, and PB1 fragments are derived from human influenza H3N2 subtype virus; NP, NS, M, PB2, and PA were derived from classical swine influenza H1N1 viruses; and PB2 and PA were originated from H9N2 avian influenza viruses. In 2007, Yao et al. reported a two-source H3N2 reassortant swine influenza virus [16]. The M and NS fragments of the strain were derived from the H1N1 swine influenza virus, whereas HA and NA were derived from H3N2 human influenza virus. In 1994, Brown et al. obtained a swine-human-avian three-source recombinant H1N2 swine influenza virus [17]. The HA gene of the strain was derived from human influenza H1N1. The NA gene was derived from the porcine H3N2 subtype, while the other six genes were originated from the H1N1 flu virus of the avian species. Karasin et al. ([6]; Karasin et al. 2002) also isolated the “swine-human-avian” triple-reassortant H1N2 swine influenza virus in the United States from 1999 to 2001. The HA, M, NP, and NS were originated from the classical H1N1 swine flu viruses, the NA and PB1 genes were from the human H3N2 influenza viruses, and the PB2 and PA genes are from the avian flu viruses.

RETRACTED

In this study, a virus was isolated from the lymph nodes and lungs of pigs suspected to be infected with swine flu viruses. Our results showed that the virus had strong pathogenicity to chick embryo and could kill the chicken embryo in 48 hours. The allantoic fluid had hemagglutination activity. It is confirmed to be a H1N2 subtype virus by HA, HI, and NA assays, electron microscopy, and whole genome sequencing and thus named A/swine/Fujian/F1/2010 (H1N2). Based on the role of pigs as intermediate hosts in the SIV interspecies transmission chain and the complexity of influenza ecology in China, it is of great importance to understand the prevalence of influenza viruses circulating in swine herds. Although EID_50_ of the isolated strains was 10^−4.6^/0.1 mL, it could infect mice and piglets without killing them, of which the isolated strains were less pathogenic.

Based on the whole genome sequencing analyses, A/Swine/Fujian/F1/2010 (H1N2) was a “swine-human-avian” reassortant virus, highly similar to A/Swine/shanghai/1/2007 (H1N2), another reassortant virus isolated in Shanghai, China. We inferred that the HA, NP, M, and NS genes were derived from the swine classical H1N1 influenza virus. The NA and PB1 genes were derived from human H3N2 subtype influenza viruses and PA and PB2 genes were from the avian influenza virus. The genetic characteristics of swine influenza virus isolation show that swine does play an important role as a “mixer” during the spread of influenza virus. Studies on the molecular and genetic evolution of swine flu are of great importance for timely detection of swine flu. The surveillance of the variation of swine influenza is critical for prevention and control of flu outbreaks.

## Figures and Tables

**Figure 1:** RT-PCR results of M gene. 1: marker 2000; 2, 3, and 4: M; 5: negative control.

**Figure 2:** Electron specular photograph of allantoic fluid after centrifugation.

**Figure 3:** RT-PCR electrophoresis of A/Swine/Fujian/F1/10 (H1N2) strain. M: marker 2000; 1 and 2: PB2; 3 and 4: PB1; 5 and 6: PA; 7 and 8: NP; 9: NS; 10: M; 11 and 12: HA; 13: NA; 14: negative control.

**Figure 4:** Phylogenetic tree based on HA nucleotide sequence.

**Figure 5:** Phylogenetic tree based on NA nucleotide sequence.

**Figure 6:** Phylogenetic tree based on PB1 nucleotide sequence.

**Figure 7:** Phylogenetic tree based on PA nucleotide sequence.

**Figure 8:** Phylogenetic tree based on PB2 nucleotide sequence.

**Figure 9:** Schematic diagram representing genes of A/Swine/Fujian/F1/2010(H1N2). The eight gene fragments were HA, NA, M, NP, NS, PA, PB1, and PB2 from top to bottom.

RETRACTED

## References

[1] Kothalawala H., Toussaint M. J. M., Gruys E. (2006). An overview of swine influenza. *Veterinary Quarterly*.

[2] Webster R. G., Bean W. J., Gorman O. T., Chambers T. M., Kawaoka Y. (1992). Evolution and ecology of influenza A viruses. *Microbiology and Molecular Biology Reviews*.

[3] Zhou N. N., Senne D. A., Landgraf J. S. (1999). Genetic reassortment of avian, swine, and human influenza A viruses in American pigs. *Journal of Virology*.

[4] Top F. H., Russell P. K. (1977). Swine influenza a at fort dix, new jersey (January–february 1976). iv. summary and speculation. *The Journal of Infectious Diseases*.

[5] Peiris J. S. M., Guan Y., Markwell D., Ghose P., Webster R. G., Shortridge K. F. (2001). Cocirculation of avian H9N2 and contemporary "human" H3N2 influenza A viruses in pigs in southeastern China: Potential for genetic reassortment?. *Journal of Virology*.

[6] Karasin A. I., Schutten M. M., Cooper L. A. (2000). Genetic characterization of H3N2 influenza viruses isolated from pigs in North America, 1977-1999: Evidence for wholly human and reassortant virus genotypes. *Virus Research*.

[7] Chang L.-Y., Shih S.-R., Shao P.-L., Huang D. T.-N., Huang L.-M. (2009). Novel Swine-origin Influenza Virus A (H1N1): The First Pandemic of the 21st Century. *Journal of the Formosan Medical Association*.

[8] Scholtissek C., Rohde W., Von Hoyningen V., Rott R. (1978). On the origin of the human influenza virus subtypes H2N2 and H3N2. *Virology*.

[9] Kawaoka Y., Krauss S., Webster R. G. (1989). Avian-to-human transmission of the PB1 gene of influenza A viruses in the 1957 and 1968 pandemics. *Journal of Virology*.

[10] Brown I. H. (2000). The epidemiology and evolution of influenza viruses in pigs. *Veterinary Microbiology*.

[11] Webby R. J., Swenson S. L., Krauss S. L., Gerrish P. J., Goyal S. M., Webster R. G. (2000). Evolution of swine H3N2 influenza viruses in the United States. *Journal of Virology*.

[12] Cong Y. L., Pu J., Liu Q. F. (2007). Antigenic and genetic characterization of H9N2 swine influenza viruses in China. *Journal of General Virology*.

[13] Zhu Q., Yang H., Chen W. (2008). A naturally occurring deletion in its NS gene contributes to the attenuation of an H5N1 swine influenza virus in chickens. *Journal of Virology*.

[14] Moreno A., Barbieri I., Sozzi E. (2009). Novel swine influenza virus subtype H3N1 in Italy. *Veterinary Microbiology*.

[15] Kundin W. D. (1970). Hong Kong A-2 influenza virus infection among swine during a human epidemic in taiwan. *Nature*.

RETRACTED

[16] Yao Y., Zhang G.-H., Liu W.-J., Chen T.-Q., Sun L. (2007). Genome sequence analysis of an H3N2 subtype swine influenza virus isolated from Guangdong province in China. *Wei sheng wu xue bao = Acta microbiologica Sinica*.

[17] Brown I. H., Chakraverty P., Harris P. A., Alexander D. J. (1995). Disease outbreaks in pigs in Great Britain due to an influenza A virus of H1N2 subtype. *Veterinary Record*.

